This article has been retracted.

# Enhanced Anti-Tumor Effect of Zoledronic Acid Combined with Temozolomide against Human Malignant Glioma Cell Expressing O^6^-Methylguanine DNA Methyltransferase

**DOI:** 10.1371/journal.pone.0104538

**Published:** 2014-08-11

**Authors:** Junya Fukai, Fumiaki Koizumi, Naoyuki Nakao

**Affiliations:** 1 Department of Neurological Surgery, Wakayama Medical University School of Medicine, Wakayama, Japan; 2 Shien-Lab, National Cancer Center Hospital, Tokyo, Japan; University of Pittsburgh, United States of America

## Abstract

Temozolomide (TMZ), a DNA methylating agent, is widely used in the adjuvant treatment of malignant gliomas. O^6^-methylguanine-DNA methyltranferase (MGMT), a DNA repair enzyme, is frequently discussed as the main factor that limits the efficacy of TMZ. Zoledronic acid (ZOL), which is clinically applied to treat cancer-induced bone diseases, appears to possess direct anti-tumor activity through apoptosis induction by inhibiting mevalonate pathway and prenylation of intracellular small G proteins. In this study, we evaluated whether ZOL can be effectively used as an adjuvant to TMZ in human malignant glioma cells that express MGMT. Malignant glioma cell lines, in which the expression of MGMT was detected, did not exhibit growth inhibition by TMZ even at a longer exposure. However, combination experiment of TMZ plus ZOL revealed that a supra-additive effect resulted in a significant decrease in cell growth. In combined TMZ/ZOL treatment, an increased apoptotic rate was apparent and significant activation of caspase-3 and cleavage of poly-(ADP-ribose) polymerase were observed compared with each single drug exposure. There were decreased amounts of Ras-GTP, MAPK and Akt phosphorylation and MGMT expression in the ZOL-treated cells. Subcutanous xenograft models showed significant decrease of tumor growth with combined TMZ/ZOL treatment. These results suggest that ZOL efficaciously inhibits activity of Ras in malignant glioma cells and potentiates TMZ-mediated cytotoxicity, inducing growth inhibition and apoptosis of malignant glioma cells that express MGMT and resistant to TMZ. Based on this work, combination of TMZ with ZOL might be a potential therapy in malignant gliomas that receive less therapeutic effects of TMZ due to cell resistance.

## Introduction

Glioblastoma multiforme (GBM) is the frequent form of malignant glioma, the most common primary brain tumor, and is characterized by poor prognosis. Stupp et al. revealed a statistically significant survival benefit for GBM patients treated with radiotherapy (RT) plus concomitant and adjuvant temozolomide (TMZ) chemotherapy, which currently represents the standard of care for newly diagnosed GBM patients [1], [2], [3]. However, despite surgery, RT and TMZ, GBM invariably recurs and ultimately leads to patients' death. To prolong tumor control and patient survival, additional therapeutic strategies are necessary.

TMZ, an oral alkylating agent, will form methyl adducts on a variety of positions on the bases of DNA [4]. Methylation of the O^6^ position of guanine (O^6^MeG) will activate mismatch repair (MMR) mechanisms and DNA damage signaling pathways, leading to G2/M cell cycle arrest and eventually to induction of cell death [4], [5], [6]. However, O^6^MeG lesions can be rapidly repaired by the cellular DNA-repair protein O^6^-methylguanine-DNA methyltransferase (MGMT) which is expressed in about 50% of GBM patients [4]. Through this mechanism, MGMT expression can cause TMZ resistance in tumor cells; otherwise, the loss of MMR system should be considered as the other mode of TMZ tolerance in GBM [7], [8]. Indeed, previous evidence analyzing GBM tissues from study patients suggests that the duration of tumor control and survival advantage conferred by TMZ chemotherapy are highly associated with the MGMT activity: active expression of MGMT predicts early tumor progression and short survival time [9], [10], [11]. Therefore, current TMZ-based adjuvant chemotherapy must be modified in order to overcome less sensitivity against malignant glioma expressing the MGMT.

Zoledronic acid (ZOL), the most potent inhibitor of bone resorption, is clinically applied to treat bone diseases of multiple myeloma or bone metastases from solid cancers because of their ability to inhibit osteoclast-mediated bone destruction. The possible mechanism of action seems to be through the mevalonate pathway by blocking the key enzyme of the post-translational prenylation of intracellular small G protein superfamily members, including small GTPases such as Ras, Rac and Rho, finally leading to apoptosis of osteoclasts [12]. Moreover, it is now becoming clear that ZOL can also affect tumor cells and exhibit direct and indirect anti-tumor effects in preclinical models: that is, anti-proliferative, proapoptotic and anti-invasive activities, and anti-angiogenic and immunomodulatory abilities [12]. On the other hand, the specific property of ZOL has attracted many researchers to look for new treatments by combining it with chemotherapeutic agents such as cisplatin, etoposide, doxorubicin and irinotecan, because such combinations have shown synergistic effects on different types of cancer cells [12].

TMZ-based adjuvant chemotherapy is a standard treatment for malignant gliomas and MGMT expression is an important predictive factor of TMZ sensitivity [1], [2], [3], [9], [10], [11]. Based on this background, there is a considerable interest in exploring new methods to efficiently suppress malignant gliomas expressing the MGMT. The use of drug combinations is a well-established principle of cancer therapy and combined therapies with TMZ will enable the potential development of new adjuvant treatments for these tumors. There are numerous reports concerning the combined effects of ZOL with anticancer agents in various cancer cell lines except for malignant gliomas [12]. ZOL has been clinically available and will be a promising candidate for a combination treatment with TMZ. In this study, we focused on ZOL as a pharmacological tool and evaluated whether ZOL can be effective as a combination drug with TMZ in human malignant glioma cells that express MGMT.

## Materials and Methods

### Ethics

This study was carried out in strict accordance with the institutional guidelines of Wakayama Medical University (WMU) Animal Care and Use Committee. The protocol was approved by the Committee on the Ethics of Animal Experiments of WMU (Permit Number: 387).

### Cell Culture

Human glioblastoma cell lines were obtained as follows: U-251 MG, T98G, SF126, A-172, AM38, and YH-13, JCRB Cell Bank (Osaka, Japan); DBTRG-05 MG, LN-229, LN-18 and M059K, ATCC (Manassas, VA). These cell lines were maintained in RPMI1640 supplemented with 10% fetal bovine serum (FBS) and cultured at 37°C in a humidified atmosphere containing 5% CO_2_.

### Chemicals

Temozolomide (TMZ) was purchased from Wako Pure Chemical (Osaka, Japan). Zoledronic acid (ZOL) (ZOMETA) was purchased from Novartis (Basel, Switzerland).

### Antibodies

Antibodies (Abs) were purchased as follows: anti-human MGMT mouse monoclonal (NeoMarker, Fremont, CA); Ras mouse monoclonal (upstate, Millipore, Temecula, CA); Akt, antiphospho-Akt, p44/42 mitogen activated protein kinase (MAPK), phospho-p44/42 MAPK, rabbit polyclonal, anti- β-actin, cleaved caspase-3, cleaved poly (ADP-ribose).

Polymerase (PARP) rabbit monoclonal, anti-mouse and rabbit IgG horseradish peroxidase-linked Abs (Cell Signaling Technology, Beverly, MA).

### Reverse Transcription-PCR

After washing twice with ice-cold PBS, 1 mL of ISOGENE (Nippongene, Toyama, Japan) reagent was added to each culture plate. Samples were removed by scraping, and stored at −80°C. Total RNA was isolated following the ISOGENE protocol as described by the manufacturer. *MGMT* mRNA expression was analyzed by reverse transcription-PCR (RT-PCR) with TaKaRa RNA PCR Kit (AMV) Ver.3.0 (TakaraBio, Shiga, Japan) also as instructed. RT-PCR for *GAPDH* served as an internal control. Bands intensities were quantified by densitometric scanning using NIH ImageJ software, readily available on the Internet. Primer sequences for human *MGMT* (624 bp) and *GAPDH* (408 bp) were 5′-ATG GAC AAG GAT TGT GAA-3′ & 5′-TCA GTT TCG GCC AGC AGG-3′ and 5′-CCC ATC ACC ATC TTC CAG GAG-3′ & 5′-AGG GAT GAT GTT CTG GAG AGC C- 3', respectively.

### Immunoblotting

Cells were lysed in lysis buffer (50 mM Hepes buffer, 1% Triton X-100, 5 mM EDTA, 50 mM sodium chloride, 10 mM sodium pyrophosphate, 50 mM sodium fluoride, 1 mM sodium orthovanadate) containing protease inhibitors (Roche Diagnostics, Penzberg, Germany). Immunoblotting were carried out, as described previously [13]. Briefly, cell lysates were fractionated by SDS-polyacrylamide gel electrophoresis. Proteins were blotted onto PVDF membranes and incubated with primary Abs, followed by probing with secondary Abs. Immunoblotted proteins were detected using the ECL Western Blotting Detection System (GE Healthcare, Buckinghamshire, UK). Bands intensities were quantified by densitometric scanning using NIH ImageJ software.

### Immunocytochemistry

Cultured cells were fixed for 20 min in 4% paraformaldehyde in PBS at room temperature (RT), blocked for 1 hour in 10% normal goat serum at RT and incubated with primary Ab overnight. Reactants were processed with the standard streptavidin-biotin immunoperoxidase method (VECTASTAIN ABC Kit, Vector, Burlingame, CA) according to the specifications of the manufacture.

Diaminobenzidine was used as the final chromogen. Immunostained cells were examined under a microscope (Keyence Biozero, Osaka, Japan).

### Growth-inhibition Assay (MTS Assay)

One thousand cells were seeded in triplicate wells of a 96-well plate in culture medium. Each concentration of chemicals was supplemented following cell adhesion. The plates were incubated for 24–168 hours at 37°C and reacted with MTS (3-[4,5-dimethylthiazol-2-yl]-5-[3-carboxymethoxyphenyl]-2-[4-sulfophenyl]-2H-tetrazolium, inner salt) reagent in the CellTiter96 Aqueous One Solution Cell Proliferation Assay (Promega Corporation, Madison, WI). MTS offers an indication of cellular proliferation status [14]. The plates were quantified by spectrophotometric reading at OD490. The percentage cell growth was calculated by comparison of the absorbance value reading obtained from treated samples *versus* controls.

### Isobologram analysis

The isobologram method of analysis is a well-known procedure for the evaluation of synergistic or antagonistic interactions between two drugs, regardless of mechanism of action of the individual drug [15]. The concentrations for TMZ and/or ZOL, required to produce the fifty percentage inhibition of growth, were obtained from its dose-response curve as determined by MTS assay. The concentrations of ZOL and TMZ are placed on the X and Y coordinates of the isobologram, respectively. The isoboles joining points representing isoeffective combinations to points on the axes representing isoeffective concentrations of each drug are all straight lines. If the data points for various dose combinations are plotted on the straight line connecting the doses of the single drugs, the combination effect can be said to be additive. Points below this line correspond to synergistic interactions, while points above the straight line indicate antagonism.

### Quantitative Analysis of Cellular Apoptosis

The cytoplasmic histone-associated DNA fragments, which are indicative of ongoing apoptosis, were quantitatively measured by using the Cell Death Detection ELISA^PLUS^ photometric enzyme immunoassay method (Roche, Inc., Mannheim, Germany) according to the manufacturer's instructions.

### Hoechst 33342/Propidium Iodide (PI) Immunofluorescence

To detect gradations of nuclear damage (DNA conformation and chromatin state), cultured cells were stained with Hoechst 33342 (Molecular Probes, invitrogen detection technologies, Eugene, OR). PI solution (DOJINDO, Kumamoto, Japan) was used for Identifying dead cells.

### Annexin V/Propidium Iodide (PI) Immunofluorescence

Redistribution of plasma membrane phosphatidyl serine is a marker of apoptosis and was assessed using Annexin-V-FLUOS (Roche Diagnostics GmbH, Mannheim, Germany), fluorescence-conjugated anticoagulant for the detection of phosphatidylserine on the outer leaflet of apoptotic cells. Cultured cells were stained with Annexin-V-Fluos and PI solution according to the manufacturer's instructions.

### Ras Pull-Down Assay

Cells were lysed with magnesium-containing lysis buffer (25 mM Hepes buffer, 150 mM sodium chloride, 1% Triton X-100, 10% glycerol, 25 mM sodium fluoride, 10 mM magnesium chloride, 1 mM EDTA, 1 mM sodium orthovanadate, 10 ug/ml leupeptin, 10 ug/ml aprotinin). Lysates were incubated with agarose-conjugate Raf-1 RBD to pull down active Ras (upstate, Millipore). The precipitates were followed by immunobotting analyses.

### In vivo xenograft assay

All surgery was performed under sodium pentobarbital anesthesia, and all efforts were made to minimize suffering. The female BALB/cA -nu/nu mice at the age of 5–6 weeks were purchased from Japan Clea (Osaka, Japan). Cells were resuspended in 200 µl of PBS and injected subcutaneously (s.c.) in the flank of mice. After a few weeks, when tumor volume had reached approximately 400–600 mm^3^, mice were randomized into four groups: control (n = 4), TMZ (n = 4), ZOL(n = 4) and TMZ/ZOL (n = 4). Groups of TMZ treatment were administered intraperitoneally (i.p.) with 10 mg/kg TMZ on DAY 1, 2, 3, 4, 5.

Groups of ZOL treatment were administered i.p. with 5 mg/kg ZOL on days 1, 3, 5 of each week for 2 weeks. Tumor volume was calculated once a week for 5 weeks (35 days) according to the following equation: tumor volume (mm^3^)  = π/6×length× (width)2; as reported previously [16]. Results are expressed as mean ± S.D.

### Statistics

Comparisons were made using unpaired Student's t test. P<0.05 was considered statistically significant.

## Results

### Expression of MGMT and chemosensitivity to TMZ in human malignant glioma cell lines

Initially, we assessed the expression of endogenous *MGMT* mRNA and protein in 10 human malignant glioma cell lines by RT-PCR and immunoblotting, respectively (Fig. 1A and B). MGMT expression was detected in three cell lines, T98G, YH-13 and LN-18, and intranuclear localization of the expressed MGMT protein was demonstrated in these cell lines by means of immunocytochemistry (Fig. 1C). Next, we evaluated chemosensitivity of malignant glioma cell lines to TMZ. T98G and LN-18 did not exhibit significant growth inhibition with less than 100 µM TMZ, as clinically achievable concentration, even at a longer exposure, whereas the 50% growth inhibition was reached at 72 hours on LN-229, in which MGMT was not expressed (Fig. 1D). These findings were consistent with the previous notion that MGMT expression could be associated with chemosensitivity of malignant gliomas to TMZ. Therefore, it is necessary to explore how to suppress MGMT-expressing malignant glioma cells, which are resistant to TMZ, in an efficient manner.

**Figure 1:** Expression of MGMT and chemosensitivity to TMZ in human malignant glioma cell lines. **A, Expression of *MGMT* gene in human malignant glioma cell lines.** RNA was isolated from ten malignant glioma cell lines. RT-PCR was done to assess *MGMT* mRNA expression. Expression of *MGMT* mRNA was detected in T98G, YH-13 and LN-18. **B, Expression of MGMT protein in human malignant glioma cell lines.** Protein extracts were prepared from ten malignant glioma cell lines. MGMT expression was analyzed by immunoblotting. β-actin was used as a loading control. Expression of MGMT protein was detected in T98G, YH-13 and LN-18. **C, Expression and localization of MGMT protein in human malignant glioma cell lines.** Cultured cells were fixed and incubated with anti-MGMT antibody. Reactants were processed with the standard streptavidin-biotin immunoperoxidase method. Diaminobenzidine was used as the final chromogen. Expression and intranuclear localization of MGMT protein was observed in T98G, YH-13and LN-18. **D, Growth-inhibitory effect of TMZ in human malignant glioma cell lines.** One thousand cells per well were placed onto a 96-well tissue culture plate and incubated overnight. TMZ was added at concentrations of 0–800 µM and incubated for 0–7 days before an MTS assay was performed. T98G and LN18 did not exhibit growth inhibition by TMZ even at a longer exposure.

### *In vitro* growth-inhibitory effect of co-treatment of ZOL with TMZ on MGMT-expressing malignant glioma cells

The use of drug combinations is a well-established principle of cancer therapy because of the perception that these drugs might act synergistically in combination. There is some preclinical evidence that the combination of ZOL with chemotherapeutic or other molecularly targeted anticancer agents may lead to an enhanced anti-tumor activity [12]. To examine whether co-treatment of ZOL with TMZ inhibits the growth of T98G and LN-18 cell lines that are resistant to TMZ, the cells were incubated in a culture medium containing TMZ (100 µM) and ZOL (40 µM) for 120 hours. As shown in Fig. 2A and B, whereas TMZ or ZOL alone did not suppress cell growth of these cell lines significantly, a combination of TMZ and ZOL markedly inhibited the growth. On the basis of this finding, we evaluated if these two agents could be synergistic in inducing cell growth inhibition of T98G. MTS assay was performed with different concentrations of ZOL in combination with TMZ at 120 hours and the resulting data were elaborated with isobologram analysis. As shown in Fig. 2C, TMZ and ZOL exerted a synergistic growth-inhibitory effect on T98G cells. Therefore, the combined use of these two agents might be an effective therapy for TMZ-resistant malignant gliomas expressing MGMT.

**Figure 2:** *In vitro* growth-inhibitory effect of co-treatment of ZOL with TMZ on MGMT-expressing malignant glioma cells. **A, Growth-inhibitory effect of ZOL in human malignant glioma T98G cell line.** One thousand cells per well were placed onto a 96-well tissue culture plate and incubated overnight. ZOL was added at concentrations of 0–80 µM and incubated for 0–5 days before an MTS assay was performed. T98G did not exhibit substantial growth inhibition by ZOL (40 µM) at 120 hours. **B, Growth-inhibitory effect of TMZ and ZOL combination in human malignant glioma cell lines.** *Upper* One thousand cells per well were placed onto a 96-well tissue culture plate and incubated overnight. TMZ (100 µM) and/or ZOL (40 µM) was added and incubated for 0–5 days before an MTS assay was performed. This figure is representative of three independent experiments. Bars, SD. *, P<0.05. *Lower* In the same experiment as *Upper*, an MTS assay after 120 hours incubation was highlighted. T98G and LN-18 exhibited significant growth inhibition by 100 µM TMZ plus 40 µM ZOL despite modest inhibition by each drug. **C, Isobologram analysis of growth-inhibitory effect of TMZ and ZOL combination in human malignant glioma T98G cell line.** Cells were treated with TMZ and/or ZOL as a single drug or in combination. Combination effect was analyzed at the 50% growth-inhibition ratio endpoints. The isobologram was based upon the dose-response curves, as determined by MTS assay. The X- and Y-axis indicate the ZOL and TMZ concentrations (µM), respectively. The isobologram plotted at the 50% endpoint was curved downward, suggesting synergistic interaction between TMZ and ZOL in T98G.

### Apoptosis-mediated cell death of MGMT-expressing malignant glioma cells by co-treatment of ZOL with TMZ

We evaluated the apoptotic effects of TMZ/ZOL combination on T98G and LN-18 cells. First, we quantitatively measured the cytoplasmic histone-associated DNA fragments, which are indicative of ongoing apoptosis (Fig. 3A). Treatment with TMZ (100 µM) and ZOL (40 µM) alone for 72 hours had a little effect on apoptosis of T98G and LN-18 cells. However, when the cells were treated with the two drugs in combination, remarkable increase of apoptosis was found. In these experimental conditions, gradations of nuclear damage and redistribution of plasma membrane phosphatidyl serine were observed at fluorescence microscopy with Hoechst33342 and Annexin-V labelling, respectively (Fig. 3B and C). Moreover, a great increase of red fluorescent cells with PI labeling was detected in the combined treatment as compared to the single treatment points (Fig. 3B). In the same experimental conditions, TMZ alone had a little effect on the activity of caspase-3 and poly (ADP-ribose) polymerase (PARP) as evaluated by immunoblotting, while ZOL alone induced a fair increase of these enzymes (Fig. 3D). Caspase-3 is one of the key executioners of apoptosis; activation of caspase-3 requires proteolytic cleavage of its inactive zymogen [17]. The nuclear enzyme PARP helps cells to maintain their viability; Cleavage of PARP facilitates cellular disassembly and serves as a marker of cells undergoing apoptosis [18]. Notably, TMZ and ZOL combination induced significant increase of the cleaved caspase-3 and PARP, suggesting that the execution of apoptosis induced by the combination played a role in the cells.

**Figure 3:** Apoptosis-mediated cell death of MGMT-expressing malignant glioma cells by co-treatment of ZOL with TMZ. **A, Apoptotic Cell Death with TMZ and ZOL combination in human malignant glioma cell lines.** Cells were treated with or without TMZ (100 µM) and/or ZOL (40 µM) for 72 hours. The cytoplasmic histone-associated DNA fragments, which are indicative of ongoing apoptosis, were quantitatively measured by using the photometric enzyme-immunoassay method. Combination of TMZ and ZOL synergistically induced apoptotic cell death in T98G and LN-18. Apoptotic response of LN-229 to TMZ (100 µM) was served as a positive control. Bars, SD. *, P<0.05. **B, Apoptotic cell death by TMZ and ZOL combination in human malignant glioma T98G cell line.** *Left* Cells were treated with TMZ (100 µM) and ZOL (40 µM) for 72 hours and stained by Hoechst 33342. Apoptosis was evidenced by chromatin margination in the cell nucleus. Scale bar represents 100 µm. *Right* Cells were treated with or without TMZ (100 µM) and/or ZOL (40 µM) for 72 hours and stained by Propidium Iodide. Cell death was more frequent in the combination treatment with Temozolomide and ZOL. Scale bar represents 100 µm. **C, Apoptotic cell death by TMZ and ZOL combination in human malignant glioma T98G cell line.** Cells were treated with TMZ (100 µM) and/or ZOL (40 µM) for 72 hours and stained by Annexin-V-FLUOS and Propidium Iodide solution. Phosphatidylserine on the outer leaflet of apoptotic cell-membranes was apparent in the combination treatment with Temozolomide and ZOL. Scale bar represents 100 µm. **D, Effect of TMZ and ZOL combination on cleavage of caspase-3 or PARP in human malignant glioma cell lines.** *Upper* Cells were treated with or without TMZ (100 µM) and/or ZOL (40 µM) for 72 hours. Expression of cleaved caspase-3 and PARP were analyzed by immunoblotting. *Lower* Relative densitometric units of the cleaved caspase-3 and PARP bands in each cell treated with or without TMZ and/or ZOL. The density of the None band is set arbitrarily at 1.0. Bars, SD. Activities of caspase-3 and PARP were prominent in the combination treatment with Temozolomide and ZOL.

### Effect of co-treatment of ZOL with TMZ on Ras activity and its downstream signaling in MGMT-expressing malignant glioma cells

Since ZOL affects the important mechanism of Ras activation [12], we evaluated the effect of ZOL treatment on Ras activity in T98G and LN-18 cell lines. In details, we studied both Ras expression and activity in the cells. ZOL (40 µM) and/or TMZ (100 µM) for 48 hours had no effect on total Ras expression levels as evaluated by immunoblotting analysis (Fig. 4A). However, ZOL alone or in combination with TMZ induced an apparent decrease of Ras activity in the cells as evaluated by affinity precipitation with raf-1 and immunoblotting analysis for Ras, although TMZ alone had no clear effect on Ras activity. These results suggest that ZOL had a direct effect on Ras activation, not on Ras expression/content. Next, we evaluated the effects of ZOL and/or TMZ on the downstream enzymes of the Ras-dependent MAPK pathway, Erk-1 and Erk-2 (Fig. 4B). ZOL alone or in combination caused a corresponding reduction of the phosphorylation of the two enzymes to Ras activity as evaluated with immunoblotting assay. On the other hand, neither the single agents nor the combination induced remarkable changes of Erk-1/2 expression. Thereafter, we evaluated the effects of the single agents or the combination on another important survival pathway, the Akt/PKB signaling at the same experimental conditions (Fig. 4C). ZOL and the combination with TMZ had an inhibitory effect on Akt phosphorylation without affecting its expression, although TMZ alone did not induce significant changes in either activity or expression of Akt.

**Figure 4:** Effect of co-treatment of ZOL with TMZ on Ras activity and its downstream signaling in MGMT-expressing malignant glioma cells. **A, Effect of TMZ and ZOL combination on Ras activity in human malignant glioma cell lines.** *Upper* Cells were treated with or without TMZ (100 µM) and/or ZOL (40 µM) for 48 hours. Active Ras GTPase was pulled down and checked by immunoblotting. Expression of Ras GTPase was also assessed using whole protein lysate. *Lower* Relative densitometric units of the Ras-GTP bands in each cell treated with or without Temozolomide and/or ZOL. The density of the None band is set arbitrarily at 1.0. Bars, SD. ZOL inhibited Ras activity in T98G and LN-18. **B, Effect of TMZ and ZOL combination on p44/42 MAPK phosphorylation in human malignant glioma cell lines.** *Upper* Cells were treated with or without TMZ (100 µM) and/or ZOL (40 µM) for 72 hours. Phospho-p44/42 MAPK was checked by immunoblotting. Expression of p44/42 MAPK was also assessed by re-blotting. *Lower* Relative densitometric units of the Phospho-p44/42 MAPK bands in each cell treated with or without TMZ and/or ZOL. The density of the None band is set arbitrarily at 1.0. Bars, SD. ZOL inhibited p44/42 MAPK phosphorylation in T98G and LN-18. **C, Effect of TMZ and ZOL combination on Akt phosphorylation in human malignant glioma cell lines.** *Upper* Cells were treated with or without TMZ (100 µM) and/or ZOL (40 µM) for 72 hours. Phospho-Akt was checked by immunoblotting. Expression of Akt was also assessed by re-blotting. *Lower* Relative densitometric units of the phospho-Akt bands in each cell treated with or without TMZ and/or ZOL. The density of the None band is set arbitrarily at 1.0. Bars, SD. ZOL inhibited Akt phosphorylation in T98G and LN-18.

### Effect of co-treatment of ZOL with TMZ on MGMT expression in MGMT-expressing malignant glioma cells

Based on the results that co-treatment of ZOL with TMZ inhibits the growth of T98G and LN-18 cell lines that are resistant to TMZ, we hypothesized that ZOL might down-regulate expression of MGMT and potentiate chemosensitivity to TMZ. Then, we analyzed MGMT expression status by RT-PCR and immunoblotting. As shown in Fig. 5A and B, both MGMT mRNA and protein levels in T98G and LN-18 cells deceased at 72 hours after treatment of ZOL alone and in combination. Thus, it is suggested that ZOL might decrease MGMT in the glioma cells and sensitize the resistant cells to TMZ.

**Figure 5:** Effect of co-treatment of ZOL with TMZ on MGMT expression in MGMT-expressing malignant glioma cells. **A, Expression of *MGMT* gene in human malignant glioma cell lines.** RNA was isolated from cells treated with or without TMZ (100 µM) and/or ZOL (40 µM) for 72 hours. *MGMT* mRNA expression was assessed by RT-PCR. *GAPDH* was used as a loading control. ZOL down-regulated *MGMT* mRNA expression in T98G and LN-18. **B, Expression of MGMT protein in human malignant glioma cell lines.** *Upper* Protein extracts were prepared from cells treated with or without TMZ (100 µM) and/or ZOL (40 µM) for 72 hours. MGMT expression was analyzed by immunoblotting. β-actin was used as a loading control. *Lower* Relative densitometric units of the Ras-GTP bands in each cell treated with or without TMZ and/or ZOL. The density of the None band is set arbitrarily at 1.0. Bars, SD. ZOL down-regulated MGMT protein expression in T98G and LN-18.

### *In vivo* growth-inhibitory effect of co-treatment of ZOL with TMZ on MGMT-expressing malignant glioma xenografts

We also investigated the effect of TMZ and ZOL combination on subcutaneous LN-18 xenografts. Tumors were allowed to grow until around 500 mm^3^, and then treatments were initiated. As shown in Fig. 6A and B, either TMZ (10 mg/kg) or ZOL (5 mg/kg) decreased the tumor growth to a mild extent, whereas a combination of TMZ and ZOL substantially enhanced the suppression of the tumor growth. Although approximate 10% body weight loss occurred in treated mice, body weight was recovered during the observation period (Fig. 6B). These results clearly show the significant *in vivo* activity of the combination treatment against the LN-18 tumor xenograft.

**Figure 6:** *In vivo* growth-inhibitory effect of co-treatment of ZOL with TMZ on MGMT-expressing malignant glioma xenografts. **A, Anti-tumor effect of TMZ and ZOL combination in human malignant glioma LN-18 cell line.** BALB/cA nude mice (female, 5–6 weeks old) bearing LN-18 tumor were separated into four treatment groups; None, TMZ, ZOL and TMZ + ZOL. TMZ (10 mg/kg) was administered i.p. on day 1, 2, 3, 4, 5. ZOL (5 mg/kg) was injected i.p. on day 1, 3, 5 of each week for 2 weeks. At day 35, combination of TMZ and ZOL apparently inhibited tumor growth of LN-18. **B, Anti-tumor effect of TMZ and ZOL combination in human malignant glioma LN-18 cell line.** *Left* BALB/cA nude mice bearing LN-18 tumor were treated with or without TMZ and/or ZOL. Tumor length and width were measured in situ with digital calipers once a week for 5 weeks (35 days). Tumor volume was calculated once a week for 5 weeks (35 days) according to the following equation: tumor volume (mm^3^)  = π/6×length× (width)^2^. Points represent mean values ± SE. Combination of TMZ and ZOL significantly inhibited tumor growth of LN-18. *Right* In the same experiment as *Left*, body weight was measured once a week for 5 weeks (35 days). Points represent mean values ± SE. Approximate 10% body weight loss occurred in treated mice, whereas body weight was recovered during the observation period.

## Discussion

Although TMZ chemotherapy is a standard of adjuvant treatment against glioblastomas, there remains to be an important problem how to control glioblastomas refractory to this therapy. Also, in our experiments, malignant glioma cells expressing MGMT were less sensitive to TMZ, as reported elsewhere [9], [10], [11]. To efficiently suppress TMZ-resistant tumors, additional therapeutic strategies are necessary and drug combination will enable the potential development of new adjuvant treatments. The present data provide evidence that ZOL efficaciously inhibits the activity of Ras and the expression of MGMT in malignant glioma cells and potentiates TMZ-mediated cytotoxicity, inducing growth inhibition and apoptosis of malignant glioma cells that express MGMT and resistant to TMZ (Fig. 7). These results suggest that combination of ZOL with TMZ therapy might be effective against malignant gliomas refractory to TMZ.

**Figure 7:** A diagram of the proposed mechanism showing anti-tumor effect of TMZ in combination with ZOL against malignant glioma cells expressing MGMT. According to the results of the present study, ZOL inhibits the activity of Ras and the expression of MGMT in malignant glioma cells and potentiates TMZ-mediated cytotoxicity, inducing growth inhibition and apoptosis of malignant glioma cells that express MGMT and resistant to TMZ. The molecular mechanism leading to the pathway indicated by the dotted arrow remains to be determined.

There are numerous reports concerning the combined effects of ZOL with anticancer agents in various cancer cell lines [12]. On different types of cancer cells, several studies have demonstrated synergistic interactions between ZOL and some commonly used chemotherapeutic drugs such as cisplatin, etoposide, doxorubicin and irinotecan [12]. However, the mechanism of synergism between ZOL and other combination drugs has not been fully discussed. In our experimental conditions, combined treatment of ZOL with TMZ resulted in enhanced anti-tumor activity on malignant glioma cells expressing MGMT. As shown in Fig. 7, there are several possible mechanisms to explain why co-treatment with ZOL leads to an inhibition of cell growth and induction of apoptosis. The simplest explanation rests in the possibility that ZOL acts as a Ras inhibitor and blocks the activation of Ras and its downstream signaling such as MAPK and Akt, which are frequently activated in malignant gliomas and suppress TMZ-induced cytotoxicity against malignant glioma cells (Fig. 4) [19], [20]. Another potentially related explanation is that ZOL itself, or through the Ras inhibition, leads to the regulation of MGMT gene expression in malignant glioma cells (Fig. 5) [21]. In any case, although the definite mechanism remains to be elucidated, co-administration of ZOL resulted in the sensitization of MGMT-expressing malignant glioma cells to TMZ. This evidence might hopefully have an impact in adjuvant chemotherapy for malignant glioma expressing MGMT.

ZOL treatment could have some merits in malignant glioma therapy.

First, malignant gliomas express elevated levels of activated Ras proteins despite the absence of activating *ras* mutations [22]. Besides, GBMs express high levels of ligand-dependent and -independent growth factor receptors such as EGFR, EGFRvIII, PDGFR, FGFR, and IGF-IR [23]. Activation of these receptors leads to tyrosine kinase activation and functional up-regulation of the Ras signaling pathway or expresses the activated form of this protein. Ras proteins are a family of membrane-associated small GTPases that transmit signals from cell surface receptors, promoting diverse cellular effects such as proliferation, survival, and angiogenesis [21], [22]. Previous studies have demonstrated that ZOL prevents a processing step necessary for membrane attachment and maturation of Ras proteins, which consequently leads to the downregulation of Ras signalling and of Akt and ERK1/2-dependent survival pathways [24]. Therefore, pharmacological blocking by ZOL can be effective in preventing activation of the Ras signaling pathway and ZOL may be of therapeutic value against malignant gliomas. Second, ZOL seems to exert anti-tumor activities against cancer cells independently of their p53 status. p53 is frequently mutated in malignant gliomas and p53 mutation status has an important role on the sensitivity of many anti-cancer drugs [25], [26]. As for TMZ, there is a report that, while malignant glioma cells with wild type of p53 experienced cell senescence or death receptor signaling-mediated apoptosis, p53-mutated glioma cells resulted in mitotic catastrophe over G2 arrest or apoptosis through mitochondrial pathway [4], [25]. ZOL, which has anti-tumor activities in spite of p53 status, is preferable for use in malignant glioma therapy [26].

There is now ample evidence from preclinical studies that not only ZOL has the ability to act directly on tumor cells of various origins, but also ZOL may exhibit indirect anti-tumor activity through anti-angiogenic and/or immunomodulatory mechanisms [12]. ZOL has been reported to reduce vascular endothelial cell and endothelial progenitor cell proliferation and migration and decrease capillary-like tube formation in vitro. Although the mechanisms by which ZOL exerts its antiangiogenic properties have not yet been clearly understood, it has been suggested that ZOL inhibits endothelial cell functions by suppression of focal adhesion assembly, inhibition of Rho geranylgeranylation and suppression of sustained activation of protein kinaseB/Akt [12]. On the other hand, ZOL has been shown to induce a significant expansion of γδ T cells, both *in vitro* and *in vivo* [12]. As opposed to antigen-recognition by conventional αβ T cells, γδ T cell-specific antigens do not need to be processed by professional antigen-presenting cells, do not require binding presentation by classical major histocompatibility complex (MHC) molecules and are therefore able to exert potent MHC-unrestricted cytotoxic effector activity toward various tumour cells including GBM [27], [28]. Although there is a main limitation investigating the anti-cancer mechanisms of ZOL i*n vivo*, since the use of immunosuppressed animals do not take into account the role of the immune system and the possible involvement of ZOL in the stimulation of an immune response, combination of ZOL could be a potent approach in anti-glioma therapy.

In our *in vivo* xenograft assay (Fig. 6), co-treatment of TMZ (10 mg/kg) and ZOL (5 mg/kg) substantially suppressed the tumor growth, although each drug decreased the tumor growth to some extent. On the other hand, we demonstrated that TMZ (100 µM) and ZOL (40 µM) exerted a synergistic growth-inhibitory effect in our *in vitro* experiments (Fig. 2). Regarding the concentration of ZOL, dose setting in the *in vivo* study may not recapitulate the *in vitro* condition; that is, ZOL concentration cannot reach to that used in vitro experiments [29]. Presumably, these results in our study suggest that the significant *in vivo* activity of the combination treatment might be due to ZOL-mediated anti-tumor effects on not only cell proliferation and induction of apoptosis but also cell adhesion, invasion, migration and VEGF production [12]. Further investigation would be needed into anti-invasive activities, and anti-angiogenic and immunomodulatory abilities of ZOL against malignant glioma in *in vitro* and *in vivo* experiments. Additionally, although co-treatment of ZOL with TMZ proved to be effective against the tumor xenograft, it remains to be elucidated whether ZOL could augment anti-tumor effect of TMZ *in vivo* as well as *in vitro*.

In chemotherapy for brain tumors including malignant glioma, it is necessary to consider whether the drug can effectively reach the tumor through the blood–brain barrier (BBB). ZOL, a small compound, could easily penetrate into the brain. However, there is some information that ZOL does not reach significant levels in the brain after intravenous administration due to a tendency to distribute the skeleton [29]. Systemic administration of ZOL would require the use of high dosage which by far exceed the clinical dosing regimens given to patients to achieve effective concentration in the brain. Therefore, when discussing the clinical relevance of ZOL therapy against malignant glioma, effective delivery of ZOL to the central nervous system may be a major point to be overcome. Regarding this problem, local administration could achieve effective concentration in the brain. For example, convection-enhanced delivery with stereotactic infusion-catheter placement would enable effective delivery of ZOL to malignant gliomas in the brain. Local administration of ZOL in the restricted environment of the brain may provide a high concentration exposure of the agent to the target cells over a limited time. The above information about drug delivery system provides us with some hope that ZOL can be used to treat patients with malignant glioma. As the next step, further investigation is needed in a clinical setting.

As shown in the Figure 2B, T98G and LN-18 exhibited significant growth inhibition by 100 µM TMZ plus 40 µM ZOL despite modest inhibition by each drug, suggesting synergistic effects of TMZ plus ZOL against malignant glioma cell lines expressing MGMT. As for LN-229, TMZ (100 µM) inhibited cell growth by more than 50% (Figure 1D and 2B). Co-treatment of TMZ and ZOL enhanced growth-inhibitory effects. Considering % cell growth inhibited by ZOL (40 µM), however, these two agents seems to be additive in inducing growth inhibition against LN-229, malignant glioma cell line that do not express MGMT. Based on the results of our MTS assays for these three cell lines (Figure 2B), ZOL (40 µM) induced growth inhibition approximately at the same level against malignant glioma cells regardless of MGMT expression status. Although inhibitory effect of cell growth by single agent ZOL was not so potent, ZOL suppressed activation of Ras and its downstream signaling in malignant glioma cells (Figure 4) as well as in other cancer cells as described in the literature [12]. Taken together, it is presumed that ZOL could exert anti-tumor activity as a Ras inhibitor against malignant glioma cells to a limited extent. However that may be, we would rather expect that ZOL can be effectively used as a combination drug with TMZ.

Expression of MGMT protein, a DNA repair enzyme, is frequently discussed as the main factor that limits the efficacy of TMZ [3], [5], [6], [7]. On the other hand, deficiency of DNA MMR proteins also contributes to TMZ resistance in GBM [7], [8]. TMZ-induced O^6^MeG, if not repaired by MGMT, mispairs with thymine during DNA replication. The resulting O^6^MeG/T mismatches are recognized by the MMR system, which triggers futile repair cycles and blocks DNA replication, leading to DNA doublestrand breaks, cell cycle arrest and eventually to cell death [5], [6]. Thus, in the absence of DNA repair by MGMT, MMR expression status influences the response of tumor cells to TMZ; that is, TMZ-induced cytotoxicity requires functional MMR and MMR deficient cells are resistant to TMZ. From this point of view in our study, ZOL-induced TMZ-mediated cytotoxicity might be attenuated against MMR deficient malignant glioma cells expressing MGMT in combination treatment of TMZ and ZOL. Further investigation is ongoing into the effect of MMR status on anti-tumor activity of TMZ and ZOL combination.

In conclusion, we have reported that ZOL cooperates and exerts enhanced cytotoxicity with TMZ against malignant glioma cells expressing MGMT and resistent to TMZ. The mechanism of synergism that we posit based on the result in the present study may be important in gliomas and warrant further examination. Because TMZ is among the most effective agents for the treatment of gliomas and TMZ can be frequently combined with other agents, the present study should prove useful in developing better TMZ-based regimens for malignant gliomas. Thus, we emphasize that combination of TMZ and ZOL using appropriate doses and schedules of administration could be a potential therapy in malignant gliomas that receive less therapeutic effects of TMZ due to cell resistance.
